RETRACTED

# Efficacy of Intermittent and Continuous Subglottic Secretion Drainage in Preventing the Risk of Ventilator-Associated Pneumonia: A Meta-Analysis of Randomized Control Trials

**DOI:** 10.3390/medicina59020283

**Published:** 2023-01-31

**Authors:** Yulis Setiya Dewi, Hidayat Arifin, Rifky Octavia Pradipta, Arina Qona’ah, Rosita Rosita, Cindy Nanda Giatin, Amel Dawod Kamel Gauda

**Affiliations:** 1 Faculty of Nursing, Universitas Airlangga, Surabaya 60115, Indonesia; 2 School of Nursing, College of Nursing, Taipei Medical University, Taipei 110, Taiwan; 3 Palembang MediRose Publisher, Palembang 30154, Indonesia; 4 Maternal and Newborn Health Nursing, College of Nursing, King Saud bin Abdulaziz University for Health Sciences (KSAU-HS), Ministry of the National Guard, Riyadh 11173, Saudi Arabia; 5 Department of Maternal and Newborn Health Nursing, Faculty of Nursing, Cairo University, Cairo 11562, Egypt

**Keywords:** intensive care unit, ventilator-associated pneumonia, subglottic secretion drainage, mechanical ventilation, health risk, infectious diseases

## Abstract

Ventilator-associated pneumonia (VAP) is hospital-acquired pneumonia that develops 48 h or longer following mechanical ventilation. However, cuff pressure fluctuates significantly due to patient or tube movement, which might result in microaspiration. Subglottic secretion drainage (SSD) has been suggested as a method for VAP prevention bundles. This systematic review and meta-analysis aims to investigate the efficacy and safety of subglottic SSD in preventing VAP. The secondary outcomes of this study are to investigate the intensive care unit (ICU) stay length and mortality rate regarding VAP. This study followed the Preferred Reporting Item for Systematic Review and Meta-Analysis guidelines. A thorough search of PubMed, Embase, and the Web of Science was conducted between June and August 2022. The study analysis used the Mantel–Haenszel method, and the quality of the included study was assessed using the Cochrane Risk of Bias 2. Eighteen randomized controlled trials with a total of 2537 intubated patients were included. It was found that SSD was associated with a lower risk of VAP (RR 1.44; 95% CI; 1.20–1.73; *p* < 0.0001). The subgroup analysis (utilizing intermittent and continuous methods) found no statistically significant difference between the two groups (*p* = 0.28). The secondary endpoints showed that there was no significant difference in mortality (RR 1.02; 95% CI; 0.87–1.20; *p* = 0.83), but there were substantial differences in ICU stays (mean difference, 3.42 days; 95% CI; 2.07–4.76; *p* < 0.00001) in favor of the SSD group. This was based on a very low certainty of evidence due to concerns linked to the risk of bias and inconsistency. The use of SSD was associated with a reduction in VAP incidence and ICU stay length, but there was no significant difference in the mortality rate.

RETRACTED

## 1. Introduction

Patients who are critically ill and frequently admitted to the intensive care unit (ICU) need invasive breathing support [1]. This invariably demands tracheal intubation to be performed to ensure free air admission. Additionally, an endotracheal cuff is wrapped around the tube’s tip to seal the extraluminal airway and enable positive pressure ventilation [1]. Incorrect regulation of cuff pressure may contribute to the difficulties associated with the use of a ventilator [2,3]. Patients in ICUs who have been on a ventilator for more than 48 h may develop ventilator-associated pneumonia (VAP) at some point [4,5]. This has significant clinical and economic implications, particularly in terms of the accompanying ICU and hospital stay length and mortality rate [6,7].

The microbial invasion of the normally sterile lower respiratory tract and lung parenchyma that leads to VAP can overcome the host’s defenses, allowing infection to spread. The aspiration of bacteria-tainted secretions that have accumulated above the endotracheal tube (ET) cuff is the most common way bacteria enter the lower respiratory tract because it is the route they take when they enter the body [5,8]. As a result, subglottic secretion drainage (SSD) is a technique that has been suggested for inclusion in VAP prevention bundles [1]. Additionally, earlier studies found that VAP was linked to greater mechanical ventilation time, longer hospital stays, consciousness issues, burns, comorbidities, prior antibiotic therapy, medication, and invasive procedures [9,10,11,12]. This study focuses on the causes of VAP due to SSD, which still lacks attention among health workers, especially nurses.

In preventing VAP, nurses have an important role during the treatment process. Regular patient monitoring and maintenance are necessary. Previous research stated that increasing the level of education would have an impact on the knowledge, attitudes, and practices of nurses in providing care and making optimal decisions [13]. However, comprehensive training on VAP is needed to increase the knowledge, compliance, and practice levels of critical care nurses [14]. Increasing the quality of care and preventing VAP can have an impact on improving patients’ quality of life [15].

Although there is a recent meta-analysis regarding the effectiveness, the number of samples and years of study are limited [16]. In addition, the meta-analysis only looked at the results of VAP prevention and mortality. This study intends to update the meta-analysis and investigate not only the ICU stay outcome but also the risk of VAP and mortality.

RETRACTED

## 2. Materials and Methods

### 2.1. Study Design

This systematic review followed the Preferred Reported Item for Systematic Review and Meta-Analysis guidelines [17]. This study has been registered in the PROSPERO with the ID registration number (CRD42022372723).

### 2.2. Eligibility Criteria

During the screening procedure, each of the articles that were discovered were categorized according to the eligibility, inclusion, and exclusion criteria that were used. The population, intervention, comparison, outcome, and study framework served as the basis for the inclusion criteria, which were as follows: (1) population: ICU patients with mechanical ventilators; (2) intervention: SSD; (3) comparison: standard care (standard ET); (4) outcome: VAP incidence, ICU stay, and mortality; (5) study: randomized controlled trials (RCTs).

In addition, studies were disregarded if they met any of the following criteria: (1) they were conducted on children; (2) the complete texts of the articles were unavailable; (3) the papers were written in a language other than English; and (4) the study did not provide total event, mean, standard deviation, and sample numbers.

### 2.3. Search Strategy

A comprehensive search of the databases MEDLINE, Embase, and the Web of Science was carried out between June and August 2022. In addition, the reference lists of pertinent publications, such as previous reviews, were carefully examined and manually screened. A comprehensive search was carried out to find all of the articles that described the use of the continuous aspiration of subglottic secretion in intubated patients or the prevention of pneumonia. Additionally, the reference lists of pertinent publications, such as prior reviews, were manually reviewed for relevance. Each scientific database’s search technique and Boolean operators are detailed in Appendix A, and the details of the literature-searching process are depicted in Figure 1.

### 2.4. Data Extraction and Quality Assessment

The primary aim was to investigate the efficacy of SSD in preventing VAP incidents. The secondary aim was to investigate the ICU stay lengths and mortality rate. Using a qualitative technique, the results were tabulated with descriptions. Information such as the author and year, study design, country of the study, participant characteristics, intervention, mean or median age, number of participants, outcome with the total event and sample data (for VAP and mortality outcome), and mean standard deviation (for ICU stays) are shown.

The final included studies were assessed for their potential for bias with the help of the revised tool for Risk of Bias in randomized trials 2, which comprises five different domains for initiative studies. The author conducted an analysis of the potential for bias using the formula that was developed by the Cochrane Collaboration. Heterogeneity was evaluated using I^2^ statistics with categories as insignificant, low, moderate, and high (cut-off limits of 0%, 25%, 50%, and 75%, respectively) [18].

RETRACTED

### 2.5. Pooled Analysis

Using the Review Manager 5.4 statistical program, a meta-analysis was conducted (Cochrane Collaboration, Oxford, UK). The dichotomous data clinical result was expressed as a risk ratio (RR) for VAP, and continuous data were expressed as a mean difference for ICU stays. An appropriate 95% confidence interval was determined.

### 2.6. Subgroup Analysis

An additional analysis—a subgroup analysis—was carried out because the studies reported different methods of SSD. The information was partitioned into intermittent and continuous groups. Following the same methodology as the prior pooled analysis, subgroups were evaluated to determine the RR for VAP incidents.

## 3. Results

### 3.1. Characteristics of Included Studies

Eighteen RCTs yielding 2537 intubated patients in the ICU were included for quantitative analysis (see Figure 1). The included studies were conducted in several locations: Turkey (*n* = 1), China (*n* = 4), Iran (*n* = 8), Belgium (*n* = 1), the United States (*n* = 1), the United Kingdom (*n* = 1), India (*n* = 1), and France and Tunisia (*n* = 1). They were published between 2012 and 2022. The mean age of participants was >36, and they were further randomized into the intervention group and control group or several follow-up intervention groups. The setting of the studies in the ICU included surgical, medical, neurological, anesthesiology ICU, and surgical-cardiac ICU. Detailed literature search procedures are presented in Table 1. Most studies’ distribution was conducted in Asian countries; therefore, this study’s conclusion is highly biased.

### 3.2. The Outcome of Included Studies

#### 3.2.1. Ventilator-Associated Pneumonia Outcomes

The results of a meta-analysis that evaluated the efficacy of SSD VAP prevention by comparing the usual care group and the SSD group are depicted in Figure 2 as a forest plot. The results indicate that there is a significant effect (*p* < 0.0001), and the RR was 1.44 (95% CI: 1.20–1.73). It was discovered that SSD could dramatically reduce VAP incidents in ICU patients with mechanical ventilation. It was also discovered that there was heterogeneity (I^2^ = 30%; *p* = 0.10).

According to the findings of the subgroup analysis, studies utilized intermittent and continuous methods in terms of both usual care and SSD intervention. The difference between the two groups was not statistically significant (*p* = 0.93). It was also discovered that there was heterogeneity (I^2^ = 0%). The results indicate that there is a significant effect between the intermittent (RR 1.54; 95% CI; 1.14–2.08; *p* = 0.0005; I^2^ = 0%) and continuous groups (RR 1.57; 95% CI; 1.19–2.07; *p* = 0.001; I^2^ = 0%). The details of the subgroup analysis are shown in Figure 3.

RETRACTED

#### 3.2.2. ICU Length of Stay Outcomes

The results of a meta-analysis that evaluated the efficacy of SSD on ICU length of stay outcomes by comparing the usual care group with the SSD group are depicted in Figure 4 as a forest plot. The results indicate that there is a significant effect (*p* < 0.00001), and the mean difference (MD) was 3.42 (95% CI: 2.07–4.76). It was discovered that SSD could dramatically reduce ICU length of stay among patients with mechanical ventilation. It was also discovered that there was heterogeneity (I^2^ = 0%; *p* = 0.45).

#### 3.2.3. Mortality Outcomes

The results of a meta-analysis that evaluated the efficacy of SSD mortality outcomes by comparing the usual care group with the SSD group are depicted in Figure 5. The results indicate that there is no significant effect (*p* = 0.31), and the RR was 1.02 (95% CI: 0.87–1.20). It was discovered that SSD had no significant effect in reducing mortality incidents in ICU patients with mechanical ventilation. It was also discovered that there was heterogeneity (I^2^ = 14%; *p* = 0.83).

### 3.3. Quality of Included Studies

Most studies had moderate to low bias as individuals, and only two studies had high biases. Figure 6 shows the risk of bias in each included study. Overall, there was no blinding, and there were differences in the baseline preventive measures used in some studies. Figure 7 shows the summary risk of bias per component assessment.

## 4. Discussion

This study conducted a meta-analysis to investigate SSD compared with the standard ET used as usual care on ICU patients who are intubated with a mechanical ventilator. The risks of VAP, ICU length of stay, and mortality were also evaluated. This study is important and provides valuable information for nurses on preventing VAP. SSD is an important indicator that needs attention from nurses who may be missing SSD events, which can cause VAP [36,37]. It was found that SSD reduced the risk of VAP and ICU length of stay but did not significantly reduce the risk of mortality. This result is consistent with previous studies that reported reductions in VAP and ICU length of stay outcomes [1,16,38,39].

RETRACTED

Ventilator-associated pneumonia is responsible for a considerable rise in the duration of mechanical ventilation, the length of stay in the ICU, the expense of that time, the need for antibiotic therapy, and patient mortality [40,41]. The accumulation of secretions in the gap between the glottis and the cuff during intubation, which cannot be removed by coughing, is the primary cause of VAP. Therefore, germs are more likely to spread throughout the lower respiratory tract [42].

In most cases, the treatment of VAP is carried out by a multidisciplinary team, including an ICU nurse [4]. When it comes to VAP, the most important thing is to lower the risk by requiring preventative practices in patient care. It is important to address all of the modifiable risk factors, one of which is endotracheal and tracheostomy suctioning through SSD equipment [4]. It is also necessary to pay attention to the observation of the cuff pressure because low cuff pressure allows bacteria to enter the body [36,43,44]. Strengthening nurses through regular training needs to be done to improve knowledge, attitude, skills, and practice levels.

The efficacy of SSD in the VAP prevention bundle has been demonstrated through this meta-analysis. The incidence of VAP was observed to be correlated with ICU length of stay in observational studies [45,46,47], and this meta-analysis suggests that SSD may decrease ICU length of stay, possibly due to a reduced risk of VAP. Guidelines for the prevention of VAP have been developed in a number of countries [48]. These guidelines urge the use of an ET that is equipped with a subglottic suctioning lumen. However, there are still certain restrictions associated with using this method. For instance, expensive specialist tubes are necessary, and the treatment is frequently followed by problems such as mucosal injury to the airway [49,50].

This highlights that the generalization of the meta-analysis is very important. This meta-analysis showed insignificant heterogeneity; it only showed moderate heterogeneity in the risk of VAP outcome and low heterogeneity in the mortality outcome. This is mirrored by a clear symmetry in the funnel plot, which may show low bias. The protocol for this study was submitted to PROSPERO to strengthen the robustness and transparency of this systematic review and meta-analysis. Furthermore, a sub-group analysis was conducted for intermittent and continuous methods to minimize the bias of this study.

However, there are some limitations to this study. First, the clinical setting in which those trials were carried out may not have been representative of the overall ICU population, as most of the studies were conducted on the Asian population. Second, some interventions caused confounding in several of the studies that were included, namely polyurethane, saline, and semi-recumbent positions. Finally, the primary problems with most of the included studies’ bias were that there was no blinding, the study authors may have had potential commercial conflicts of interest, there were differences in the baseline preventive measures that were applied, there was a potentially high level of heterogeneity as a result of differences in methodology between studies, and there were differences in the devices used for SSD.

RETRACTED

Based on this meta-analysis, there is moderate evidence that SSD can be used as an intervention in preventing VAP. SSD is one of several interventions in the VAP prevention bundle, including the administration of antibiotics [51]. However, adverse events, especially tracheal mucosal injury due to SSD administration, need to be considered. This meta-analysis did not observe an adverse event related to the administration of SSD, so a further meta-analysis is expected to add to these outcomes. In addition, adverse events and risk of death between intermittent and continuous methods were not observed in this meta-analysis because many of the included studies did not report the SSD method used or combined analysis of both in one group study.

## 5. Conclusions

Subglottic secretion drainage has a reasonable amount of evidence supporting its usage as an intervention for the prevention of VAP. Moreover, SSD could reduce ICU length of stay but not the mortality rate. However, further studies are required to compare intermittent and continuous SSD, and more high-quality research is needed to determine SSD’s potential role in medical care. Furthermore, a study to evaluate the co-effectiveness of SSD usage needs to be conducted.

## Figures and Tables

**Figure 1:** Preferred Reported Item for Systematic Review and Meta-Analysis flow diagram.

**Figure 2:** Risk of VAP in the usual care group vs. the SSD group.

**Figure 3:** Subgroup analysis of VAP risk outcome between the usual care group and the SSD group [25,32].

**Figure 4:** ICU length of stay in the usual care group vs. the SSD group.

**Figure 5:** Mortality in the usual care group vs. the SSD group.

**Figure 6:** Traffic light plot risk of bias.

**Figure 7:** Summary of risk of bias.

**Table 1:** Characteristics of included studies.

Study	Design	Location	Setting	Age (Mean SD)	Gender (Male %)	Intervention of Treatment Group	Method of SSD
Akdogan et al. (2017) [19]	RCT	Turkey	Anesthesiology ICU	IG: 60.32 (21.55) CG: 61.34 (19.78)	IG: 28 (75.68) CG: 52 (54.17)	Endotracheal tube with subglottic drainage and cuff pressure monitorization	Continuous
Chai et al. (2022) [20]	RCT	China	ICU	-	CG: 24 (40%) IG: 28 (46.66%)	suction with 0.9% normal saline with 5% inhaled eucalyptus	-
Chen et al. (2016) [21]	RCT	China	ICU	IG: 51.8 (12.0) CG: 51.8 (12.1)	IG: 16 CG: 25	subglottic secretion drainage	-
Chow et al. (2012) [22]	Pilot RCT	Iran	Surgical ICU	IG: 70.3 (14.3) CG: 79.4 (12.5)	56	SSD with the saliva ejector tube	Continuous
Damas et al. (2015) [23]	RCT	Belgium	ICU	IG: 66 (55–75) CG: 65 (55–75)	IG: 107 CG: 127	Subglottic secretion suctioning	-
Deem et al. (2016) [24]	Pilot RCT	USA	ICU	IG: 55 (17) CG: 53 (16)	10	Polyurethane-cuffed tube equipped with a port for continuous aspiration of subglottic secretions (PUC-CASS-ETT)	Continuous
Gopal et al. (2015) [25]	RCT	UK	Surgical and Cardiac ICU	IG: 72.4 (8.2) CG: 72.1 (7.4)	*n* = 699	SSD with Venner- PneuX tube	Intermittent
Jena et al. (2016) [26]	Pilot RCT	India	Neurological ICU	IG: 36.9 (12.8) CG: 42.2 (17.9)	32	Suction above cuff endotracheal tube (SACETT)	-
Mahmoodpoor et al. (2013) [27]	RCT	Iran	Surgical ICU	IG: 54.00 (19.49) CG: 55.71 (19.39)	67.2	Taperguard- Polyurethane cuff with the continuous aspiration of subglottic secretions	-
Mahmoodpoor et al. (2013) [27]	RCT	Iran	Surgical ICU	IG: 57.31 (19.77) CG: 55.71 (19.39)	64	Sealguard- Polyurethane cuff with continuous aspiration of subglottic secretions	-
Mahmoodpoor et al. (2017) [28]	A prospective randomized trial	Iran	ICU	IG: 54.0 (19.2) CG: 54.5 (18.1)	IG: 102 CG: 84	Evac tube	Intermitten
Mahmoodpoor et al. (2020) [29]	RCT	Iran	ICU	55	72.8	Polyurethane cuff with continuous aspiration of subglottic secretions	-
Mansoor et al. (2016) [30]	RCT	Iran	ICU	IG: 38.24 (24.71) CG: 43.35 (24.71)	IG: 27 CG: 19	Endotracheal tube with subglottic suction port (Mallinckrodt™ TaperGuard Evac Oral Tracheal Tube; Covidien, Mexico)	Intermittent
Naghibi et al. (2019) [31]	A randomized, double-blind, placebo-controlled trial	Iran	ICU	IG: 38 (14) CG: 45.57 (14.53)	IG: 10 CG: 9	SSD with sodium chloride	Intermittent
Philippart et al. (2015)-a [32]	A multicenter, prospective, open-label RCT	France and Tunisia	medical-surgical ICUs	65.6 (53.0–77.2)	IG: 83 CG: 92	PVC, Cylindrical	Continuous
Philippart et al. (2015)-b [32]	a multicenter, prospective, open-label RCT	France and Tunisia	medical-surgical ICUs	63.2 (53.4–76.4)	IG: 91 CG: 96	PVC, Conical	Continuous
Seyfi et al. (2013) [33]	RCT	Iran	ICU	-	-	SSD	-
Tao et al. (2014) [34]	RCT	China	ICU	-	-	SSD	Intermittent and continuous
Qiao et al. (2018) [35]	RCT	China	ICU	IG: 65.1 (5.6) CG: 64.6 (7.6)	IG: 25 CG: 23	Bronchoscopic sputum suction	Continuous

RETRACTED

## Data Availability

Not applicable.

## Appendix A

*PubMed*

#1 ((“ventilated”[All Fields] OR “ventilates”[All Fields] OR “ventilating”[All Fields] OR “ventilation”[MeSH Terms] OR “ventilation”[All Fields] OR “ventilate”[All Fields] OR “ventilations”[All Fields] OR “ventilator s”[All Fields] OR “ventilators, mechanical”[MeSH Terms] OR (“ventilators”[All Fields] AND “mechanical”[All Fields]) OR “mechanical ventilators”[All Fields] OR “ventilator”[All Fields] OR “ventilators”[All Fields] OR “ventillation”[All Fields])

#2 ((“subglottal”[All Fields] OR “subglottic”[All Fields]) AND (“suction”[MeSH Terms] OR “suction”[All Fields] OR (“mechanical”[All Fields] AND “aspiration”[All Fields]) OR “mechanical aspiration”[All Fields]))

#3 (“pneumonia, ventilator associated”[MeSH Terms] OR (“pneumonia”[All Fields] AND “ventilator associated”[All Fields]) OR “ventilator-associated pneumonia”[All Fields] OR (“ventilator”[All Fields] AND “associated”[All Fields] AND “pneumonia”[All Fields]) OR “ventilator associated pneumonia”[All Fields]))

*Embase:*

#1 “subglottic mechanical aspiration” OR “subglottic mechanical suction” OR “mechanical aspiration” OR suction OR subglottic

#2 “ventilator-associated pneumonia” OR “ventilator associated pneumonia” OR pneumonia

*Web of Science*

#1 ((((ALL=(Ventilator-Associated Pneumonia)) OR ALL=(Pneumonia)) OR ALL=(Respiratory Tract Infections)) OR ALL=(Healthcare-Associated Pneumonia)) OR ALL=(Hospital Acquired Pneumonia)

#2 (((((ALL=(Mechanical Aspiration)) OR ALL=(Suction)) OR ALL=(mucus)) OR ALL=(secretion)) OR ALL=(secret)) OR ALL=(subglottic)
